# DNA Binding and Photocleavage Studies of Cobalt(III) Polypyridine Complexes: [Co(en)_2_PIP]^3+^, [Co(en)_2_IP]^3+^, and [Co(en)_2_phen-dione]^3+^

This article has been retracted.

**DOI:** 10.1155/2007/54562

**Published:** 2007-06-25

**Authors:** Penumaka Nagababu, S. Satyanarayana

**Affiliations:** Department of Chemistry, Osmania University, Hyderabad 500 007, Andhra Pradesh, India

## Abstract

In this paper, three complexes of type [Co(en)_2_PIP]^3+^(PIP=2-phenylimidazo[4,5-f][1,10,] phenanthroline)(1), [Co(en)_2_IP]^3+^ (IP = imidazo[4,5-f][1,10,] phenanthroline)(2), and [Co(en)_2_phen-dione]^3+^(1,10 phenanthroline 5,6,dione)(3) have been synthesized and characterized by UV/VIS, IR, ^1^H NMR spectral methods. Absorption spectroscopy, emission spectroscopy, viscosity measurements, and DNA melting techniques have been used for investigating the binding of these two complexes with calf thymus DNA, and photocleavage studies were used for investigating these binding of these complexes with plasmid DNA. The spectroscopic studies together with viscosity measurements and DNA melting studies support that complexes 1 and 2 bind to CT DNA (= calf thymus DNA) by intercalation mode via IP or PIP into the base pairs of DNA, and complex 3 is binding as groove mode. Complex 1 binds more avidly to CT DNA than 2 and 3 which is consistent with the extended planar ring *π* system of PIP. Noticeably, the two complexes have been found to be efficient photosensitisers for strand scissions in plasmid DNA.

## 1. INTRODUCTION

The interaction of transition metal complexes with DNA has been extensively studied in the past few years. Metal complexes of the type [M(LL)_3_]^n+^ where LL is either 1,10,phenathroline or modified phenanthroline ligand are particularly attractive species to recognize and cleavage DNA [1–4]. Barton demonstrated that tris(phenanthroline) complexes of ruthenium(II) display enantiomeric selectivity in binding to DNA, which can be served as spectroscopic probes in solution to distinguish right- and left-handed DNA helies [5]. The ligands or the metal in these complexes can be varied in an easily controlled manner to facilitate an individual application. The change in the metal ion or ligand would lead to changes in the binding mode and affinity [6, 7]. Much attention has been paid to the complexes of Ru(II) [8–10]. We choose to concentrate our work on cobalt(III) ethylenediamine polypyridyl complexes which have the same interesting characteristics and DNA cleaving properties as Ru(II) complexes. We have chosen ethylenediamine because in classical antitumor agent (cis platin) one of the ligands must be N donor and possessing at least one hydrogen atom attached to nitrogen.

In this paper, we report the synthesis and characterization of the two complexes 1 and 2 (see Schemes 1 and 2), and their binding ability to CT DNA, DNA-binding properties are studied by electronic absorption, luminescent spectra, viscosity measurement, and DNA melting curve. The photochemical DNA cleavages of the complexes are also demonstrated.

## 2. EXPERIMENTAL METHODS

### 2.1. Materials

All materials were purchased and used without further purification unless otherwise noted. The compounds 1,10 phenanthroline-5,6-dione [11], (IP) and (PIP) [12], [Co(en)_2_phen]Br_3_ [13] *cis*-[Co(en)_2_Cl_2_]Cl · 3H_2_O [14], and [Co(en)_2_L]Br_3_ were prepared by the procedure given below. The absorption spectra of CoCl_2_ 6H_2_O, *cis* [Co(en)_2_Cl_2_]Cl, and [Co(en)_2_PIP]Br_3_ are shown in Figure 1. All the experiments involving the interaction of the complexes with DNA were carried out in buffer (5 mM tris-HCl, 50 mM NaCl, pH 7.2). A solution of CT DNA in the buffer gave a ratio of UV absorbance at 260 and 280 nm of about 1.90 indicating that the DNA was sufficiently free of protein [15]. The DNA concentration per nucleotide was determined by absorption spectroscopy using the molar absorption coefficient (6600 M^−1^Cm^−1^) at 260 nm [16].

## 3. SYNTHESIS OF COMPLEXES

### 3.1. [Co(en)_2_PIP]Br_3_

A mixture of *cis*-[Co(en)_2_Cl_2_]Cl (1.43 g) and phenylimi-dazo[4,5-f][1,10,] phenanthroline (1 g) was dissolved in EtOH (6 ml) and NaBr (3.0 g) in H_2_O (5 ml) was added and heated on a water bath until a dark yellow solution was formed. It was then cooled in ice where the thick crystalline precipitate of [Co(en)_2_PIP]^3+^ was collected and recrystallized from water (30 ml). The yield by this method was about 80% (Mol. Wt 715). (Elemental analysis found: C, 37.12; H, 3.2; N, 15. Calc. for C_23_N_8_H_28_Br_3_Co : C, 38.63; H, 3.95; N, 15.67.) IR stretching frequencies are (C=C); 1458, (C=N); 1508, (Co–N (en)); 779, (Co–N(ligand)); 625.5.

### 3.2. [Co(en)_2_IP]Br_3_

The complex [Co(en)_2_IP]^3+^ was prepared according the procedure described above from the mixture of *cis*-[Co(en)_2_-Cl_2_]Cl (1.43 g) and IP (1 g). (Yield: 88%.) (Elemental analysis found: C, 37.28; H, 3.2; N, 15.6. Calc. for C_23_N_8_H_28_-Br_3_Co: C, 38.63; H, 3.95; N, 15.67.) IR stretching frequencies are (C=C); 1398, (C=N); 1558, (Co–N (en)); 614, (Co–N(ligand)); 573.

### 3.3. [Co(en)_2_phen-dione]Br_3_

The complex [Co(en)_2_phen-dione]^3+^ was prepared according to the procedure described above from the mixture of *cis*-[Co(en)_2_Cl_2_]Cl (1.43 g) and phen-dione (1 g). (Yield: 88%.) IR stretching frequencies are (C=C); 1384, (C=N); 1559, (Co–N (en)); 626, (Co–N(ligand)); 615. (Elemental analysis found: H 3.3 C 30. N 13.1 O. Calc. for, C_16_N_6_O_2_H_22_Br_3_Co H, 3.53, C, 30.55, N, 13.36.)

## 4. PHYSICAL MEASUREMENTS

### 4.1. Elemental analysis and conductivity data

Carbon, hydrogen, and nitrogen analyses were obtained from microanalytical Heraeus Carlo Etba 1108 elemental analyser. Chloride analysis was done. The metal contents were estimated from these solutions on atomic absorption spectrometer Perkin-Elmer 23380. The conductivity of metal complexes was measured in freshly prepared DMSO solutions using digital conductivity bridge (model: DI-909) and a dip-type cell calibrated with KCl solution.

## 5. SPECTRAL ANALYSIS

UV/visible spectra were recorded with Elico bio-spectro-photometer, model BL198, IR spectra were recorded on a Hitachi U-3410, KBr phase on Perkin-Elmer FTIR-1605 spectrophotometer, ^1^H NMR spectra were measured on a Varian XL-300 MHz spectrometer with D_2_O as a solvent at room temperature and tetramethylsilane (TMS) as the internal standard, magnetic susceptibility measurements for solid samples of the complexes were carried out using Faraday bakany model. Hg [Co(CNS)_4_] were employed as magnetic susceptibility standards, microanalyses (C, H, and N) were carried out on a Perkin-Elmer 240 of elemental analyzer. For the absorption spectra an equal solution of DNA was added to both complex solutions and reference solution to eliminate the absorbance of DNA itself.

Viscosity experiments were carried out using an Ostwald viscometer maintained at a constant temperature at 30.0 ± 0.1°C in athermostatic water bath. Calf thymus DNA samples approximately 200 base pairs in average length were prepared by sonicating in order to minimize complexities arising from DNA flexibility [17]. Data were presented as (*η*/*η*_0_)^1/3^ versus the concentration of Co(III) complexes, where *η* is the viscosity of DNA in presence of complex, *η*_0_ is the viscosity of DNA alone. Viscosity values were calculated from the observed flow time of DNA-containing solutions (*t* > 100 s) corrected for the flow time of buffer alone (*t*_0_)*η* = (*t − t*_0_)/*t*_0_, where *t* is the observed flow time of DNA and *t*_0_ is the flow time of buffer [18]. The DNA melting experiments were carried by controlling the temperature of the sample cell with a Shimadzu circulating bath while monitoring the absorbance at 260 nm. For the gel electrophoresis experiments, super coiled pBR 322 DNA (100 *μ*M) was treated with Co(III) complexes in 50 mM Tris-HCl, 18 mM NaCl buffer, pH = 7.2, and the solution was incubated for 1 hour in the dark, then irradiated at room temperature with a UV lamp (302 nm, at 10 W). The samples were analyzed by electrophoresis for 2.5 hour at 40 V on a 0.8% agarose gel in Tris acetic acid EDTA buffer; pH 7.2. The gel was stained with 1 *μ*g/ml ethidium bromide and then photographed under UV light.

## 6. SPECTROSCOPIC CHARACTERIZATION

The IR spectral data for the complexes were determined; two complexes clearly exhibit a band at 1450 and 1560–1590 cm^−1^, corresponding to C=C and C=N of the ring, respectively. Bands at around 626 and 579 cm^−1^ corresponding to Co–N (en) and Co–N of (L=PIP, IP and phen-dione) NH_2_ (en) bending at around 1650 cm^−1^ were observed. The UV-visible spectral peaks were observed at 317, 492, 347, 437 nm and fluorescence peaks at 407, 408, and 609 of 1, 2, and 3 complexes, respectively, based on the literatures data on the spectral properties of complexes 2 and 1. Bands appearing in the spectra of Co(III) complexes can be assigned exclusively to MLCT charge transition bands between 400–500 nm, Table 1, [19]. The electronic environment of many aromatic hydrogen atoms (PIP, IP, and phen-dione) are similar and hence their ^1^H NMR spectra appear in a narrow chemical shift range. In fact the aromatic regions of the spectra of these complexes are complicated due to the overlapping of several signals, which have precluded the identification of individual resonance. In the ^1^H NMR spectra of the cobalt(III) complexes the peaks due to various H-atoms of PIP, IP, and phen-dione were shifted downfield compared to the free ligands suggesting complexation in Figure 1. As expected the signal for PIP, IP, and phen-dione appeared in the range between 7.5 to 9.2 ppm in agreement with an earlier report [19], CH_2_ groups of the ethylenediamine gave peaks at 2.72, (4H, en-CH_2_) and 3.0, (2H, en-CH_2_).

## 7. RESULTS AND DISCUSSION

### 7.1. Absorption spectral studies

The application of electronic absorption spectroscopy is one of the most useful techniques for DNA binding studies [20]. Complex binding with DNA through intercalation usually results in hypochromism and bathchromism, due to the intercalative mode involving a strong stacking interaction between an aromatic chromophore and the base pairs of DNA. The extent of the hypochromism commonly parallels the intercalative binding strength. The absorption spectra of complexes 1, 2, and 3 in absence and presence of CT DNA are given in Figures 2, 3, and 4. As the concentration of DNA is increased, it results in hypochromism and moderate bathochromic shift in the UV-visible spectra of three complexes 1, 2, and 3. According to the data presented in Figures 1, 2, and 3, it seems that the change in absorption spectra of the two complexes upon addition of DNA follows: 1 > 2 > 3. These spectral data may suggest a mode of binding that involves a stacking interaction between the complex and the base pairs of DNA. To compare quantitatively the binding strength of the two complexes, the intrinsic binding constants *K* of the two complexes with CT DNA were determined according to the following equation [21] through a plot of [DNA]/∑b−∑f) versus [DNA]

(1) $$\frac{\left[\text{DNA}\right]}{\sum_{a}-\sum_{f}}=\frac{\left[\text{DNA}\right]}{\left(\sum_{b}-\sum_{f}\right)}+\frac{1}{\left[K\left(\sum_{b}-\sum_{f}\right)\right]},$$

where [DNA] is the concentration of DNA in base pairs, the apparent absorption coefficients ∑_*a*_, ∑_*f*_, and ∑_*b*_ correspond to *A*_obsd_/[Co], the extinction coefficient for the free cobalt complex and the extinction coefficient for the free cobalt complex in the fully bound form, respectively. In plots [DNA]/(∑_*b*_ − ∑_*f*_) versus [DNA], *K* is given by the ratio of slope to intercept. Intrinsic binding constants *K* of 1, 2, and 3 were obtained about 5.34 ± 0.2 × 10^4^, 4.575 ± 0.3 × 10^4^, and 3.9 ± 0.1 × 10^4^ M^−1^ from the decay of the absorbance. The binding constants indicate that complex 1 binds strongly than 2 > 3. This result is expected, since PIP possesses a greater planar area and extended *π* system than that of IP which will lead to PIP penetrating more deeply into and makes stacking more strongly. Hypochromism was indeed observed in the complexes with the order being 1 > 2 > 3.

### 7.2. Fluorescence studies

The complexes 1, 2, and 3 can emit luminescence in Tris buffer (pH 7.0) at ambient temperature with maxima at 408, 407, and 609 nm. Binding of both complexes to DNA was found to increase the fluorescence intensity. The emission spectra of both complexes in the absence and presence of CT DNA are shown in Figures 5, 6, and 7. The plots of the relative intensity versus the ratio of [DNA]/[Co] are also inserted in Figures 5, 6, and 7. Upon addition of CT DNA, the emission intensity increases steadily. The emission intensity difference between absence of CT DNA and presence of CT DNA is greater for PIP complex than IP and phen-dione complex as shown in Figures 5, 6, and 7. The extent of enhancement increases on going from 3 to 2 to 1 and which is consistent with the above absorption spectra results. The order of increase in emission intensity of complexes is 1 > 2 > 3. These results were strengthened by viscosity studies.

This observation is further supported by the emission quenching experiments using [Fe(CN)_6_]^4−^ as quencher. The method essentially consists of titrating a given amount of DNA binding-metal complexes with increasing the concentration of [Fe(CN)_6_]^4−^ and measuring the change in fluorescence intensity. The ion [Fe(CN)_6_]^4−^ has been shown to be able to distinguish differentially bound Cobalt(III) complexes. The positively charged free complex ions should be readily quenched by [Fe(CN)_6_]^4−^, where as DNA bound cobalt complex is protected from the quencher, because highly negatively charged [Fe(CN)_6_]^4−^ would be repelled by the negatively change DNA phosphate backbone. The ferro-cyanide quenching curves for 1, 2, and 3 in the presence and absence of CT DNA are shown in Figure 8. Obviously complex 1 inserts into DNA much deeper than complexes 2 and 3. The absorption and fluorescence spectroscopy studies thus determine the binding of complexes with DNA.

### 7.3. Viscosity studies

The mode of the two complexes binding to DNA was explained by viscosity measurements. Optical photo-physical probes are necessary, but do not give sufficient clues to support a binding model. Hydrodynamic measurements that are sensitive to length change (i.e., viscosity and sedimentation) are regarded as the least ambiguous [18]. For complexes 2 and 1 the viscosity of DNA increases highly with the increasing of the concentration of complex which is similar to that of proven intercaltor EtBr [22]. Both complexes change the relative viscosity of DNA in a manner consistent with binding by intercalation mode shown in Figure 9. This result also parallels the pronounced hypochromism and spectral red shift and emission enhancement of both complexes, whereas this result is comparable with proven classical intercalator EtBr. Viscosity of DNA increases with the increase of the concentration of EtBr. So these two complexes increase DNA helix length. On the basis of the viscosity results, it shows that complexes bind with DNA through intercalation mode. The order of increase in viscosity of complexes follows the order 1 > 2 > 3.

### 7.4. DNA melting studies

Another strong evidence for binding of the complexes 1, 2, and 3 to the double helix of DNA is the melting temperature *T_m_*. The binding of small molecules into the double helix is known to increase the helix melting temperature. Helix melting temperature is the temperature at which the double helix is denatured into single-stranded DNA. The extinction coefficient of DNA bases at 260 nm in the double-helical form is much less than in the single stranded form. Hence melting of the helix leads to an increase in the absorption at this wavelength. Thus the transition temperature from helix to coil can be determined by monitoring the absorbance of the DNA base at 260 nm as a function of temperature. The melting curves of CT DNA in the absence and presence of 1, 2, and 3 are presented in Figure 10. The increase in the melting temperature values of IP and PIP comparable to the value observed (Table 2) with the classical intercalators EtBr. It is clear from these figures that the complexes 1 and 2 are intercalator because the relative absorbance is so high compared to that of the pure DNA sample. The increase in absorbance of complexes follows the order 1 > 2 > 3.

## 8. PHOTOACTIVATED CLEAVAGE OF pBR 322 DNA BY COMPLEXES

There has been considerable interest in DNA endonucleolytic cleavage reactions that are activated by metal ions [23, 24]. The delivery of high concentrations of metal ion to the helix, in locally generating oxygen or hydroxide radicals, leads to an efficient DNA cleavage reaction. DNA cleavage was monitored by relation of supercoiled circular pBR 322 (form I) into nicked circular (form II) and linear (form III). When circular plasimd DNA is subjected to electrophoresis, relatively fast migration will be observed for the supercoiled form (form I). If scission occurs on one strand (nicking), the supercoils will relax to generate a slower-moving open circular form (form II) [25]. If both strands are cleaved, a linear form (form III) will be generated that migrates between forms I and II. Figure 11 shows the gel electrophoretic separations of plasmid pBR 322 DNA after incubation with Co(III) complexes and irradiation at 302 nm. Figure 9 reveals the conversion of Form I and II after 60 min irradiation in the presence of varying concentrations of 1, 2, and 3. It was observed that by increasing the concentration of 1, 2, and 3, form (I) slightly diminishes gradually. The same has been observed with increasing irradiation time. This is the result of single stranded cleavage of pBR322 DNA. It can also be seen in Figure 11 that neither irradiation of DNA at 302 nm without Co(III) nor incubation with Co(III) without light yields significant strand scission. It is most likely that the reduction of Co(III) is the important step leading to DNA cleavage. Further studies are required to find out the path of reaction mechanism.

## 9. CONCLUSIONS

The binding behavior of complexes 1, 2, and 3 with DNA was characterized by absorption titration, fluorescence quenching, and viscosity measurements. The results show that the binding constants followed the order: 1 > 2 > 3 which is consistent with the extended planar and *π* system of PIP.

## Figures and Tables

**Figure 1:** Absorption spectra of CoCl_2_6H_2_O (1), *cis* [Co(en)_2_Cl_2_]Cl (2), and [Co(en)_2_L]Br_3_ (3).

**Scheme 1:** 

**Scheme 2:** 

**Scheme 3:** 

**Figure 2:** Absorption spectra of [Co(en)_2_PIP]^3+^ in the absence and presence of CT DNA in Tris-HCl buffer. The absorbance changes upon increasing CT DNA concentrations. (10 *μ*L, 20 *μ*L, 30 *μ*L, 40 *μ*L—of DNA addition), [Co] = 10 *μ*M, [DNA] = 0–126 *μ*M. The arrows show the decrease in intensity up on increasing DNA concentration. Insert: plots of [DNA]/(Σ*a* − Σ*f*) versus [DNA] for the titration of DNA with Co(III) complex.

**Figure 3:** Absorption spectra of [Co(en)_2_IP]^3+^ in the absence and presence of CT DNA in Tris-HCl buffer in the absence (top) absorbance decreases upon increasing CT DNA concentrations, (10 *μ*L, 20 *μ*L, 30 *μ*L, 40 *μ*L—of DNA addition), [Co] = 10 *μ*L, [DNA] = 0–126 *μ*L. The arrows show the decrease in intensity up on increasing DNA concentration. Insert: plots of [DNA]/(Σ*a* − Σ*f*) versus [DNA] for the titration of DNA with Co(III) complex.

**Figure 4:** Absorption spectra of [Co(en)_2_phen-dione]^3+^ in the absence and presence of CT DNA in Tris-HCl buffer, in the absence (top) absorbance changes upon increasing CT DNA concentrations. (10 *μ*L, 20 *μ*L, 30 *μ*L, 40 *μ*L—of DNA addition), [Co] = 10 *μ*M, [DNA] = 0–126 *μ*M. The arrows show the intensity decrease up on increasing DNA concentration. Insert: plots of [DNA]/(Σ*a* − Σ*f*) versus [DNA] for the titration of DNA with Co(III) complex.

**Figure 5:** Emission spectra of complex of [Co(en)_2_PIP]^3+^ in aqueous buffer (Tris 5 mM, pH 7.2) at 298 K in the presence of CT DNA. [Co] = 20 *μ*M, [DNA]/[Co] 0, 5, 10 …. λ_mex_ = 407 nm. Arrow shows the intensity change upon increasing DNA concentrations. Insert: plots of relative integrated emission intensity versus [DNA]/[Co].

**Figure 6:** Emission spectra of complex of [Co(en)_2_IP]^3+^ in aqueous buffer (Tris 5 mM, pH 7.2) at 298 K in the presence of CT DNA. [Co] = 20 *μ*M, [DNA]/[Co] 0, 5, 10 …. λ_mex_ = 408 nm. Arrow shows the intensity change upon increasing DNA concentrations. Insert: plots of relative integrated emission intensity versus [DNA]/[Co].

**Figure 7:** Emission spectra of complex of [Co(en)_2_phen-dione]^3+^ in aqueous buffer (Tris 5 mM, pH 7.2) at 298 K in the presence of CT DNA. [Co] = 20 *μ*M, [DNA]/[Co] 0, 5, 10 …. λ _mex_ = 608 nm. Arrow shows the intensity change upon increasing DNA concentrations. Insert: plots of relative integrated emission intensity versus [DNA]/[Co].

**Figure 8:** Emission quenching curves of (A) [Co(en)_2_phen-dione]^3+^ in presence of DNA (▪), (B) [Co(en)_2_IP]^3+^ (▴) and (C) [Co(en)_2_PIP]^3+^ (⧫) alone ([Co] = 2 *μ*mol/cm^−3^, [DNA]/[Co] = 40).

**Figure 9:** Effect of increasing amount of [Co(en)_2_PIP]^3+^ (A), [Co(en)_2_IP]^3+^ (B), and [Co(en)_2_phen-dione]^3+^ (C) on the relative viscosities of CT DNA at 25 ± 0.1°C.

**Figure 10:** Thermal melting curves of calf thymus DNA alone and in presence of complexes [Co(en)_2_PIP]^3+^ (a), [Co(en)_2_IP]^3+^ (b), and [Co(en)_2_phen-dione]^3+^ (c).

**Figure 11:** Photoactivated cleavage of pBR 322 DNA, lane 1 control plasmid DNA (untreated pBR 322), lanes 2–5 addition of complex 5 *μ*L, 10 *μ*L, 20 *μ*L, 30 *μ*L, and 6th lane +5 *μ*L at 0 time lanes 7, 8 +5 *μ*L complex upon irradiation (λ_irrd_ = 302 nm) at 5 minutes, 10 minutes, complex (A) [Co(en)_2_phen-dione]^3+^, (B) [Co(en)_2_IP]^3+^, and (C) [Co(en)_2_PIP]^3+^.

**Table 1:** λ_max_ for different complexes.

Complexes	Peak	Peak

CoCl_2_6H_2_O	229	492 nm
*cis* [Co(en)_2_Cl_2_]Cl	346	594 nm
[Co(en)_2_PIP]Br_3_	317	495 nm
[Co(en)_2_IP]Br_3_	347	453 nm
[Co(en)_2_phen-dione]Br_3_	333	445 nm

**Table 2:** Thermal melting temperature (Tm) for CT DNA and CT DNA + various complexes.

Compound	T_*M*_°C

CT DNA	60
[Co(en)_2_phen]^3+^	62
[Co(en)_2_IP]^3+^	64
[Co(en)_2_PIP]^3+^	68

## ABBREVIATIONS

CT DNA: Calf thymus DNA
PIP: 2-phenylimidazo[4,5-f][1,10,]phenanthroline
IP: Imidazo[4,5-f][1,10,]phenanthroline
Phen: [1,10,]phenanthroline
en: ethylenediamine
EtBr: Ethedium bromide.

## References

[1] Sigman DS (1986). Nuclease activity of 1,10-phenanthroline-copper ion. *Accounts of Chemical Research*.

[2] Sigman DS, Mazumder A, Perrin DM (1993). Chemical nucleases. *Chemical Reviews*.

[3] Jenkins Y, Friedman AE, Turro NJ, Barton JK (1992). Characterization of dipyridophenazine complexes of ruthenium(II): the light switch effect as a function of nucleic acid sequence and conformation. *Biochemistry*.

[4] Carlson DL, Huchital DH, Mantilla EJ, Sheardy RD, Murphy WR (1993). A new class of DNA metallobinders showing spectator ligand size selectivity: binding of ligand-bridged bimetallic complexes of Ru(II) to calf thymus DNA. *Journal of the American Chemical Society*.

[5] Barton JK (1983). Tris (phenanthroline) metal complexes: probes for DNA helicity. *Journal of Biomolecular Structure & Dynamics*.

[6] Barton JK (1986). Metals and DNA: molecular left-handed complements. *Science*.

[7] Carter MT, Rodriguez M, Bard AJ (1989). Voltammetric studies of the interaction of metal chelates with DNA. 2. Tris-chelated complexes of cobalt(III) and iron(II) with 1,10-phenanthroline and 2,2′-bipyridine. *Journal of the American Chemical Society*.

[8] Morgan RJ, Chatterjee S, Baker AD, Strekas TC (1991). Effects of ligand planarity and peripheral charge on intercalative binding of Ru(2,2′-bipyridine)_2_L^2+^ to calf thymus DNA. *Inorganic Chemistry*.

[9] Sitlani A, Long EC, Pyle AM, Barton JK (1992). DNA photocleavage by phenanthrenequinone diimine complexes of rhodium(III): shape-selective recognition and reaction. *Journal of the American Chemical Society*.

[10] Nagababu P, Latha JNL, Satyanarayana S (2006). DNA-binding studies of mixed-ligand (ethylenediamine)ruthenium(II) complexes. *Chemistry and Biodiversity*.

[11] Yamada M, Tanaka Y, Yoshimoto Y, Kuroda S, Shimao I (1992). Synthesis and properties of diamino-substituted dipyrido [3,2-*α*: 2′, 3′ -*c*]phenazine. *Bulletin of the Chemical Society of Japan*.

[12] Wu J-Z, Ye B-H, Wang L (1997). Bis(2,2′-bipyridine)ruthenium(II) complexes with imidazo[4,5-f][1,10]-phenanthroline or 2-phenylimidazo[4,5-f][1,10]phenanthroline. *Journal of the Chemical Society—Dalton Transactions*.

[13] Barve AC, Ghosh S, Kumbhar AA, Kumbhar AS, Puranik VG (2005). DNA-binding studies of mixed ligand cobalt(III) complexes. *Transition Metal Chemistry*.

[14] Bailar JC, Fernelius WC (1946). Cis & trans dichlorobis - (ethylenediamine) Co (III) chloride. *Inorganic Syntheses: Volume II*.

[15] Marmur J (1961). A procedure for the isolation of deoxyribonucleic acid from microorganisms. *Journal of Molecular Biology*.

[16] Reichmann ME, Rice SA, Thomas CA, Doty P (1954). A further examination of the molecular weight and size of desoxypentose nucleic acid. *Journal of the American Chemical Society*.

[17] Chaires JB, Dattagupta N, Crothers DM (1982). Studies on interaction of anthracycline antibiotics and deoxyribonucleic acid: equilibrium binding studies on interaction of daunomycin with deoxyribonucleic acid. *Biochemistry*.

[18] Satyanaryana S, Dabrowiak JC, Chaires JB (1993). Tris(phenanthroline)ruthenium(II) enantiomer interactions with DNA: mode and specificity of binding. *Biochemistry*.

[19] Barton JK (1986). Metals and DNA: molecular left-handed complements. *Science*.

[20] Barton JK, Danishefsky AT, Goldberg JM (1984). Tris(phenanthroline)ruthenium(II): stereoselectivity in binding to DNA. *Journal of the American Chemical Society*.

[21] Wolfe A, Shimer GH, Meehan T (1987). Polycyclic aromatic hydrocarbons physically intercalate into duplex regions of denatured DNA. *Biochemistry*.

[22] Zhang Q-L, Liu J-G, Chao H, Xue G-Q, Ji L-N (2001). DNA-binding and photocleavage studies of cobalt(III) polypyridyl complexes: [Co(phen)_2_IP]^3+^ and [Co(phen)_2_PIP]^3+^. *Journal of Inorganic Biochemistry*.

[23] Hertzberg RP, Dervan PB (1982). Cleavage of double helical DNA by (methidiumpropyl-EDTA)iron(II). *Journal of the American Chemical Society*.

[24] Graham DR, Marshall LE, Reich KA, Sigman DS (1980). Cleavage of DNA by coordination complexes. Superoxide formation in the oxidation of 1,10-phenanthroline-cuprous complexes by oxygen-relevance to DNA-cleavage reaction. *Journal of the American Chemical Society*.

[25] Barton JK, Raphael AL (1984). Photoactivated stereospecific cleavage of double-helical DNA by cobalt(III) complexes. *Journal of the American Chemical Society*.

